# Prevalence of pulmonary hypertension and its associated factors among chronic obstructive pulmonary diseases patients at public hospitals of Addis Ababa, Ethiopia, 2024: a facility-based cross-sectional study

**DOI:** 10.3389/fpubh.2024.1456235

**Published:** 2024-11-26

**Authors:** Tsehaynew Kasse, Amanuel Elias, Arega Abebe Lonsako, Yalemzer Agegnehu

**Affiliations:** College of Medicine and Health Sciences, Arba Minch University, Arba Minch, Ethiopia

**Keywords:** pulmonary hypertension, chronic obstructive pulmonary disease, adults, Addis Ababa, Ethiopia

## Abstract

**Background:**

Pulmonary hypertension (PH) is a serious medical condition characterized by elevated pressure in the lung blood vessels, with chronic heart and lung diseases being the most common causes worldwide. However, there is a dearth of studies on the prevalence of pulmonary hypertension and its associated factors among chronic obstructive pulmonary disease (COPD) patients in Ethiopia and the study area.

**Objective:**

This study aimed to assess the prevalence of pulmonary hypertension and its associated factors among patients with chronic obstructive pulmonary disease at public hospitals in Addis Ababa, Ethiopia, 2024.

**Methods:**

A facility-based cross-sectional study involving 422 COPD patients charted in Addis Ababa town, Ethiopia from May – June 2024 was conducted. Respondents’ records were chosen using simple random numbers. Structured, and pretested questionnaires, were used to collect data. The data were coded and entered into EpiData 3.1 before being exported to SPSS version 25 for analysis. Logistic regression was employed to identify factors influencing the prevalence of pulmonary hypertension. Statistical significance was set at *p* < 0.05 with a 95% confidence interval.

**Results:**

The study found the prevalence of pulmonary hypertension was 52% (95% CI: 49, 54.4%). Aged above 55 years [Adjusted Odds Ratio (AOR): 2.45 (1.55–3.9), Being male (AOR): 2.5 (1.5–4.1)]. Furthermore, having a history of alcohol [(AOR): 5.5 (2.4–13)], a history of smoking [(AOR): 4.6 (2.7–7.8), and congestive heart failure (AOR): 2.65 (1.5–4.6)], all increase the likelihood of pulmonary hypertension.

**Conclusion:**

The study revealed a higher prevalence of pulmonary hypertension among COPD patients. Significant associations were found with being male, belonging to an older age group, and having a history of alcohol use, smoking, and congestive heart disease. Implementing screening programs, smoking cessation programs, educational initiatives, and counseling patients on lifestyle modifications were recommended.

## Introduction

Pulmonary hypertension (PHN) is a medical condition characterized by elevated pressure within the blood vessels of the lung (1), specifically 20 mmHg and above of mean arterial pressure (2). Approximately 1% of the population is estimated to be affected by pulmonary hypertension of which 80% are estimated to be in the developing world (3). As the gold standard method, right heart catheterization is an invasive procedure, the widely practiced method for diagnosing PHN is Transthoracic Doppler Echocardiography (4–6) which is also true for Ethiopia (7).

Unfortunately, according to the WHO report of 2023, more than 90% of COPD deaths occur in low and middle-income countries. Chronic obstructive pulmonary disease is a lung disease characterized by a persistent reduction of airflow with no cure (8).

Patients with PHN exhibit general symptoms such as dyspnea, weakness, chest pain, and cough (4). A study in Ethiopia among HIV patients with PHN found that exertional dyspnea, cough, and leg swelling were the most commonly observed symptoms (7).

The most common cause of PHN is chronic heart and lung diseases worldwide (3, 9). This is similar in Africa, as a study across the continent in 2016 showed that about 69 and 11% of PHN cases were caused by left heart disease and lung disease, respectively (10). A systematic review and meta-analysis in Africa in 2022 revealed that almost 63% of pulmonary hypertension is caused by chronic obstructive pulmonary disease (COPD) (11).

Unfortunately, according to the WHO report of 2023, more than 90% of COPD deaths occur in low and middle-income countries. Chronic obstructive pulmonary disease is a lung disease characterized by a persistent reduction of airflow with no cure (8).

The development of pulmonary hypertension during COPD has disastrous consequences such as decreased exercise tolerance, increased hospitalization rate, and higher mortality rate (4, 5, 12). A retrospective study in Denmark (13) shows that the 5-year survival rate of COPD patients with PHN was 37%, while it was 63% among non-PH patients.

Pulmonary hypertension is a rising issue with more attention recently, and low-income countries need to give more emphasis and recognition (3). A study in sub-Saharan Africa in 2019 (14), stated a limitation of literature on risk factors of PH in sub-Saharan Africa.

To the extent of the investigator’s knowledge, no study assesses PH prevalence and factors among COPD patients in Ethiopia. Therefore, this study aims to assess the prevalence of PH and associated factors among COPD patients in Addis Ababa, Ethiopia. Therefore, this study aims to assess the prevalence of PH and associated factors among COPD patients in Addis Ababa, Ethiopia.

## Methods and materials

### Study design and study period

An institution-based cross-sectional study was conducted from May to June 2024.

### Study area/setting

The study was conducted in Addis Ababa, the capital city of Ethiopia, with an estimated population size of 5,703,628 in 2024 (15). Addis Ababa is the 4th Highest Capital in the world. Located at the foot of Mount Entoto, at an altitude of 2,355 meters above sea level. According to the data obtained from Addis Ababa City Administration Health Bureau, there are 13 public hospitals in Addis Ababa, which were giving different services to the public. Four hospitals (Tikur Anbessa Specialized Hospital, Zewditu Memorial Hospital, St. Paulo’s Hospital, and Ras Desta Hospital were randomly selected to be the target public hospitals). 400, 210, 300, and 190 COPD patients visited Tiku Anbesa Specialized Hospital, Zewditu Memorial Hospital, St. Paulos Hospital, and Ras Desta Hospital, respectively, last year, making a total of 1,100 COPD.

### Source population and study population

#### Source of population

The source population was COPD patients who were treated from 2019 to 2023.

#### Study population

The study population was all randomly selected COPD patients who were from 2019–2023.

### Inclusion and exclusion criteria

#### Inclusion criteria

All COPD patients who had been treated in the selected hospitals in the last year were included in the study.

#### Exclusion criteria

All COPD patients who had been treated in the selected hospitals in the last year but did not have complete medical records were included in the study.

### Sample size determination and sampling technique

The sample size of the study was determined using the single population proportion formula. Taking into account a 95% confidence interval (CI) and a 5% margin of error (d), along with accounting for a prevalence rate of 50% for the prevalence of pulmonary hypertension among COPD patients in Ethiopia, due to no previous studies, and considering a 10% non-response rate, the final sample size was 422.

### Sampling technique/procedure

A random sampling technique was employed to select four hospitals. The sample size was proportionally allocated to each hospital based on the total number of COPD patients visited in the last year before data collection. The total number of COPD patients (N) was determined (1,100). A proportional allocation factor (Nh) was calculated (n/N). This factor (0.384) was multiplied by the number of COPD patients in each hospital (ni) to determine the sample size allocated to each hospital (nh). To select the required sample, in each hospital, simple random sampling technique was used (Figure 1).

**Figure 1:** Schematic representation of the sampling procedure of COPD patients visiting the selected public hospitals in Addis Ababa, Ethiopia, 2024.

### Operational definition

#### Pulmonary hypertension

Pulmonary hypertension is a type of high blood pressure that affects the arteries in the lungs and the right side of the heart. Pulmonary hypertension (PH) is a disease with significant morbidity and mortality. At the time of this study, PH is defined as an elevated mean arterial pressure (mPAP) of ≥20 mmHg at rest, although the diagnosis of PH is made by Doppler echocardiography or right heart catheterization (RHC) (16, 17).

#### COPD

A common lung condition known as chronic obstructive pulmonary disease (COPD) is characterized by restricted airways that cause severe breathing difficulties. Previous research has shown a connection between the pathophysiology of COPD and the inflammatory infiltration of leukocytes in the airway. Chronic obstructive pulmonary disease (COPD) is a persistent and progressive respiratory disorder characterized by expiratory airflow limitation caused by chronic inflammation. Evidence has shown that COPD is correlated with neutrophil chemotaxis toward the airways, resulting in neutrophilic airway inflammation (18).

#### Cigarette smoking

A COPD who smokes at least one cigarette per day for at least 12 months before the study (19).

#### Alcohol drinker

COPD who drinks three or more times a week for at least 12 months of the period before the study (20).

#### Chat chewing

Khat chewing within the past month he or she will be classified as a current chewer, had a history of chewing classified as a former chewer otherwise classified as never chewer (21, 22).

### Data collection procedure and tool

The data were collected using a secondary data collection method (chart review pretested questions) based on a questionnaire adapted from prior studies. The first portion contains questions regarding the research participants’ socio-demographic traits, followed by health-related and behavioral aspects, and the internal consistency of items was found to be a Cronbach alpha value of 0.8. Four BSc Nurses will gather data, and two supervisors will be involved, supervisors will be involved and have daily on-site supervision till the end of the data collection period. Data collectors and supervisors will be trained for 2 days on research ethics, instruments, and data collection practices, as well as on the questionnaire. A pretest will also be administered.

### Data processing and analysis

After the data was collected, it was coded and entered into Epi-Data version 3.1 and then exported to the SPSS version 26 statistical package for further analysis. The data was re-coded and cleaned. Descriptive and summary statistics such as frequency, percentage, mean, and standard deviation were used to describe the different variables. Figures and tables were used to summarize the results.

Multi-collinearity between independent variables was checked for all candidate variables with variable inflation factor (VIF) scores with the values (1.4–2.5). Bivariable logistic regression analysis was conducted between each independent variable and dependent variable. A crude odds ratio (COR) along with a 95% confidence interval (CI) was used to present the results of the bivariable analysis. All variables with association in bivariable analysis at *p*-value ≤0.25 were entered into a multivariable logistic regression model to assess the adjusted association between dependent and independent variables. The adjusted odds ratio (AOR) along with a 95% CI and *p*-value <0.05 was used to determine the strength of the association and to declare statistical significance in the final model. The Hosmer-Lemeshow goodness of fit test was used to check model fitness with the value (0.45). Finally, the final results were presented using appropriate means such as texts, tables, and figures.

### Data quality control

A pre-test of 5% of the total sample size was conducted to assess the questionnaire’s appropriateness, and medical registration of the questionnaire items before data collection at St Peter Specialized Hospital, which is not included in the study. Following the pretest, all data collectors and supervisors were given training on the study’s goal and how to obtain necessary data. Supervision was provided by the supervisors and Principal Investigator. At the end of each data collection day, the investigator checked for completeness or fulfillment of the quality of the recorded information.

## Results

### Socio-demographic characteristics of study participants

This study involved a total of 422 adult patients whose charts were reviewed, resulting in a 100% response rate. The participants were predominantly male (64.7%) and married (88.9%), with half of them falling in the 56–80 years age group (52.6%). A majority of the respondents were government employees (58.8%) and urban residents (63.4%). Nearly one-third of the participants (29.6%) were unable to read and write. The mean age of the participants was 54.15 years with a standard deviation of ±10.96 (Table 1).

**Table 1:** Socio-demographic characteristics of COPD patients visiting public hospitals hospital of Addis Ababa, Ethiopia, 2024.

Variable	Category	Frequency	Percentage
Age	<56 years	200	47.4
	56–80 years	222	52.6
Sex	Female	149	35.3
	Male	273	64.7
Marital status	Single	18	4.3
	Married	375	88.9
	Windowed	13	3.1
	Divorced	16	3.8
Educational status	No formal education	125	29.6
	Primary education	120	28.4
	Secondary	103	24.4
	Above secondary	74	17.3
Occupation	Housewife	70	16.6
	Government employee	248	58.8
	Daily labor	36	8.5
	Merchant	28	6.6
	Private employee	40	9.5
Residence	Urban	269	63.7
	Rural	15	36.7

### Behavioral-related characteristics of study participants

The study revealed that 28.2% of the respondents had a history of smoking, with 54% of them reporting less than 1 year. In terms of alcohol consumption, 11.4% (48) of the participants had a history of alcohol intake, and more than half (52.7%) reported less than 1 year. Additionally, less than 5% (4.3%) of the respondents had a history of chewing chat, and among them, 83.3% reported less than 1 year (Table 2).

**Table 2:** Behavioral-related characteristics of COPD patients visiting public hospitals hospital of Addis Ababa, Ethiopia, 2024.

Categories	Frequency	Percent
History of alcohol intake	Yes = 48	11.4
	No = 374	88.6
Duration of drinking alcohol	<1 year = 25	52.7
	1–5 years = 23	47.3
History of smoking	Yes = 119	28.2
	No = 303	71.8
Duration of smoking	<1 year = 62	54
	1 and above year = 57	46
History of chewing	Yes = 18	4.3
	No = 404	95.7
Duration of chewing	<1 year = 15	83.3
	1 and above years = 3	16.7

### Clinical comorbidity characteristics of study participants

In the reviewed charts of respondents, we found notable comorbidities that may influence the prevalence of diseases. Specifically, approximately 13.3% (56 individuals) were identified as HIV positive, while around 24% (100 individuals) were diagnosed with congestive heart failure (Table 3).

**Table 3:** Clinical comorbidity characteristics of COPD patients visiting public hospitals hospital of Addis Ababa, Ethiopia, 2024.

Variable	Category	Frequency	Percent
History of HIV/AIDS	No	366	86.7
	Yes	56	13.3
History of CHF	No	322	76.3
	Yes	100	23.7

CHF, Congestive Heart Failure; HIV/AIDS, Human Immune Virus/Acquired Immune Deficiency Syndrome.

### Prevalence of pulmonary hypertension

The study found that among 422 COPD adult patients, 220 (52%) had pulmonary hypertension, with a 95% confidence interval of 49.6 to 54.4% (Figure 2). The majority (58.6%) had moderate pulmonary hypertension, while 35.9% had mild and only 5% had severe pulmonary hypertension. Regarding the duration of diagnosis, the study found that 44.5% were diagnosed within 1–5 years, 39.5% were diagnosed within the first year of visit, 10.9% were diagnosed between 5 and 10 years, and 5% were diagnosed for more than 10 years.

**Figure 2:** Prevalence of pulmonary hypertension among COPD adult patients visiting public hospitals hospital in Addis Ababa, Ethiopia, 2024.

### Factors associated with the prevalence of pulmonary hypertension

A total of eleven variables were analyzed to identify factors significantly associated with the prevalence of pulmonary hypertension. Factors such as age, sex, educational level, having a history of alcohol, history of smoking, and congestive heart failure were statistically significant at a *p*-value less than 0.25 in bivariable analysis. However, in the multivariable analysis, age, sex, history of alcohol intake, history of smoking, and presence of congestive heart failure were found to be statistically significant at a *p*-value less than 0.05 (Table 4).

**Table 4:** Factors associated with the prevalence of pulmonary hypertension among COPD adult patients visiting public hospitals hospital in Addis Ababa, Ethiopia, 2024.

Variable	Categories	Pulmonary hypertension		COR (95% CI)	AOR = (95% CI)	*p*-value
		Yes (%)	No (%)			
Age	<56 years	127 (63.5%)	73 (36.5%)	1	1	
	56–80 years	93 (41.9%)	129 (58.1%)	2.41 (1.63–5.57)	2.45 (1.55–3.9)**	<0.01
Sex	Female	96 (64.4%)	53 (35.6%)	1	1	
	Male	124 (45.4)	149 (54.6%)	2.18 (1.4–3.3)	2.5 (1.5–4.1)**	<0.01
Educational status	No formal education	62 (49.6%)	63 (50.4%)	1.07 (0.6–1.9)	1.4 (0.65–2.84)	0.42
	Primary	64 (53.3%)	56 (46.7%)	0.92 (0.5–1.65)	1.23 (0.59–2.56)	0.58
	Secondary	56 (54.4%)	47 (45.6%)	0.89 (0.49–1.61)	1.02 (0.48–2.2)	0.95
	Above secondary	38 (51.4%)	36 (48.6%)	1	1	
History of alcohol intake	Yes	9 (18.8%)	39 (81.3%)	5.6 (2.6–11.9)	5.5 (2.4–13)**	<0.01
	No	211 (56.4%)	163 (43.6%)	1	1	
History of smoking	Yes	30 (25.2%)	89 (74.8%)	4.9 (3.1–8.01)	4.6 (2.7–7.8)**	
	No	113 (37.3%)	190 (62.7%)	1	1	
History of CHF	Yes	33 (33%)	67 (67%)	2.81 (1.75–4.5)	2.65 (1.5–4.6)**	0.001
	No	187 (58.1%)	135 (41.9%)	1	1	

*p < 0.05, **p < 0.01; CHF, Congestive Heart Failure.

The study found that respondents aged 55 years and older were approximately three times more likely to develop pulmonary hypertension compared to those aged 55 and below [Adjusted odds ratio; 2.45 (1.55–3.9)]. Similarly, male respondents had higher odds of developing pulmonary hypertension compared to their female counterparts [AOR: 2.5 (1.5–4.1)]. Furthermore, having a history of alcohol use increased the odds of pulmonary hypertension by about sixfold [AOR: 5.5 (2.4–13)] compared to not having it. Having a history of smoking also increased the odds by nearly five times [AOR: 4.6 (2.7–7.8)] when compared to their non-smoking counterparts, and having congestive heart failure tripled the likelihood of pulmonary hypertension [AOR: 2.65 (1.5–4.6)] compared to those who did not have congestive heart failure.

## Discussion

The study found the prevalence of pulmonary hypertension was 52% (95% CI, 49, 54.4%), with factors such as age, sex of respondents, history of alcohol use, smoking, and congestive heart disease increasing the likelihood of developing this condition.

The prevalence of pulmonary hypertension in this study aligns with previous research conducted in Africa (49–74.7%) (11) as reported in a meta-analysis and systematic review. However, it was lower compared to studies from Europe (23.3–37.6%) (23), China (39.2%) (24), and India (16%) (25). This variation could be attributed to differences in study settings, periods, socioeconomic status, and access to healthcare services. Comparably, a large proportion of respondents in this study were rural dwellers, which may have influenced the prevalence rate.

Furthermore, the prevalence in this study was lower than that reported in Pakistan (75.5%) (26). This difference could be explained by the fact that the altitude in Pakistan is about three times higher than in Ethiopia, and altitude has been associated with an increase in pulmonary hypertension.

Regarding factors associated with the prevalence of pulmonary hypertension, the study found that respondents aged 55 years and older were approximately three times more likely to develop pulmonary hypertension compared to those aged 55 and below. This finding was in agreement with studies conducted in Pakistan (26), and the Netherlands (6), the possible justification could be primarily due to cardiovascular changes and a higher prevalence of comorbidities due to aging such as COPD, age-related left ventricular diastolic dysfunction, and portal hypertension.

Similarly, male respondents had higher odds of developing pulmonary hypertension compared to their female counterparts. The findings were found to be supported by a study conducted in Italy (27). A possible reason could be hormonal differences in that females have higher levels of estrogen, which has a protective effect against the development of pulmonary hypertension (28), and men are more likely to smoke and be exposed to occupational hazards compared to women.

Furthermore, having a history of alcohol use increased the odds of pulmonary hypertension by about sixfold compared to not having it. The findings were in agreement with a study conducted in Sweden (29), possibly, it could be attributed to several factors, including alcohol’s impact on the cardiovascular system, its pro-inflammatory effects, and its ability to induce oxidative stress.

Having a history of smoking also increased the odds of pulmonary hypertension by nearly five times when compared to their non-smoking counterparts, which is supported by studies conducted in Europe (30), and the USA (31). The possible justification could include direct vasoconstrictive effects, chronic inflammation, oxidative stress, hypoxic pulmonary vasoconstriction, of nicotine and other chemicals in cigarettes. Furthermore having congestive heart failure tripled the likelihood of pulmonary hypertension compared to those who did not have congestive heart failure, which is concurrent with studies conducted in Denmark (13) and Nigeria (32). The possible reason could primarily be due to the backward transmission of increased left atrial pressure, neurohormonal activation and remodeling, increased blood volume, thromboembolic disease, and hypoxemia-induced hypoxic pulmonary vasoconstriction (33).

## Conclusion

The prevalence of pulmonary hypertension among COPD patients in this study was higher. Being male, older age group, having a history of alcohol use, smoking, and congestive heart disease were found to increase the likelihood of pulmonary hypertension.

### Recommendations

Based on the study findings, several recommendations are proposed to enhance the management of pulmonary hypertension among COPD patients, particularly by integrating our new insights into existing knowledge.

Firstly, the town health office should implement targeted programs aimed at reducing the prevalence of pulmonary hypertension specifically among COPD patients. This includes establishing screening programs, health education, and promotion campaigns that differentiate between age groups specifically those under 56 years and those aged 56–80 years.

For younger patients (< 56 years), the screening program could focus on identifying early signs of pulmonary hypertension and providing education on lifestyle modifications, including smoking cessation and alcohol use awareness. For older patients (56–80 years), the program should include more comprehensive evaluations for comorbidities and tailored interventions that address the complexities of managing multiple health conditions.

Secondly, health professionals should routinely screen all COPD patients for signs of pulmonary hypertension, with an emphasis on age-specific risk factors. Counseling should be adapted to each age group, ensuring that younger patients receive guidance on prevention and lifestyle changes, while older patients are provided with strategies to manage their overall health and quality of life. A special focus should be given for health failure patients with close follow-up and preventive measures for pulmonary hypertension.

Lastly, further research is recommended to conduct large-scale clinical trials and longitudinal studies that not only explore the natural history of pulmonary hypertension among COPD patients but also examine how these variables (factors) impact quality of life and mortality outcomes over time.

### Strength and limitation of the study

Strengths: The study’s ability to offer an accurate snapshot of the prevalence within this particular population without requiring long-term follow-up. Limitations: The cross-sectional design of this study limits the ability to establish causal relationships between the dependent and independent variables. Additionally, the sample had a significantly higher proportion of male participants compared to females, which may affect the generalizability of the prevalence rates observed. Furthermore, the reliance on secondary data analysis raises concerns regarding specificity, data accuracy, contextual information, and completeness.

## Data Availability

The raw data supporting the conclusions of this article will be made available by the authors, without undue reservation.
